# Research on Public Administration and Resource Allocation Based on Blockchain and Structured Occupational Therapy

This article has been retracted.

**DOI:** 10.1155/2022/2623656

**Published:** 2022-06-11

**Authors:** Qiyou Zhu

**Affiliations:** School of Law, Anhui Normal University, Wuhu, Anhui 241002, China

## Abstract

In order to explore the public administration and resource allocation based on blockchain and structured occupational therapy, this paper takes the public affairs in the prevention and control of the Corona Virus Disease 2019 (COVID-19) epidemic as an example to conduct research. On the basis of summarizing and analyzing the previous published literatures, this study expounded the research status and significance of public administration and resource allocations; elaborated the development background, current status and future challenges of blockchain, and structured occupational therapy; introduced the methods and principles of data quality collaboration model and multiparty collaboration standard management; analyzed the case background of public administration and resource allocation in the prevention and control of the COVID-19 epidemic; discussed the public administration mechanism based on blockchain and structured occupational therapy; established a resource allocation method based on blockchain and structured occupational therapy; fathomed the role of the distributed ledger established by blockchain to increase the information symmetry of public administration activities; proposed a blockchain-established special machine trust for resource allocation; and finally, anatomized the data security sharing and access control mechanism based on blockchain and structured occupational therapy. The research results show that the public administration and resource allocation in this paper can effectively realize the data integration of the whole process and all departments and show the whole data and realize the traceability of the whole process. The blockchain revolutionizes the hierarchical leadership method of traditional resource allocation, shortens the distance between superiors and subordinates, makes information dissemination more fluent, and handles things more efficiently, making resource allocation ultimately form a flatter organization structure. In the original trust system of resource allocation, the blockchain and structured occupational therapy realizes the reconstruction of the trust system by preventing information tampering, using information encryption technology, and using information traceability technology. The results of this paper provide a reference for further research on the public administration and resource allocation based on blockchain and structured occupational therapy.

## 1. Introduction

The institutional design of public administration participation includes the disclosure of public administration affairs, the improvement of participation channels, the promotion of community autonomy, and the formulation of relevant participation laws. Through these efforts, more and better information sources, participation tools, participation carriers, and legal guarantees can be provided for resource allocation and participation in urban public administration [1]. Implementing the disclosure of public administration affairs means that all public administration affairs should be made public except those involving social security or state secrets that are not allowed to be disclosed by law. This kind of disclosure includes not only the disclosure of decision-making activities and their processes in public administration activities but also the disclosure of relevant documents, materials, and information and intelligence formulated in public administration [2]. The disclosure of public administration affairs provides necessary relevant information for resource allocation and participation in urban public administration and is the basis for ensuring the enthusiasm of public administration of resource allocation [3]. In urban public administration, the independence of civil society should be cultivated first, and institutional guarantees should be provided for the healthy development of this social body. Therefore, it has a corresponding legal activity space to cultivate diversified social interest groups and enable resource allocation expresses its political interests and requirements in the participation of urban public administration, so that modern urban public administration activities will be full of vigor and vitality [4].

Blockchain technology is a data structure that links data blocks in chronological order and uses cryptographic algorithms to ensure that the data stored in this way cannot be tampered with and cannot be forged and can be easily verified. The use value of blockchain is that organizations can track ledgers, and organizations can jointly create, develop, and track an immutable history of transactions and determine continuous events [5]. As the core content of the new technology revolution, blockchain is a new generation of technological innovation after the Internet, which has application advantages such as decentralization, immutability, traceability, security, and transparency. As a distributed system, blockchain requires a negotiation process relative to the information stored by each node at runtime [6]. Compared with the advantages of high anti-interference and fast response speed of distributed systems, distributed systems have the problem that it is difficult to reach a consensus in the network. The immutability of distributed system information is based on the immutability of the consensus established through negotiation [7]. An attacker cannot change the consensus established in the system by attacking a few nodes. The negotiation process will cause the information storage speed to be slower than the centralized system, and it is necessary to ensure that the negotiation results of normal nodes will not produce inconsistent results due to the interference of malicious nodes [8].

In order to explore the public administration and resource allocation based on blockchain and structured occupational therapy, this paper takes the public affairs in the prevention and control of the Corona Virus Disease 2019 (COVID-19) epidemic as an example to conduct research. On the basis of summarizing and analyzing the previous published literatures, this study expounded the research status and significance of public administration and resource allocations; elaborated the development background, current status and future challenges of blockchain, and structured occupational therapy; introduced the methods and principles of data quality collaboration model and multiparty collaboration standard management; analyzed the case background of public administration and resource allocation in the prevention and control of the COVID-19 epidemic; discussed the public administration mechanism based on blockchain and structured occupational therapy; established a resource allocation method based on blockchain and structured occupational therapy; fathomed the role of the distributed ledger established by blockchain to increase the information symmetry of public administration activities; proposed a blockchain-established special machine trust for resource allocation; and finally, anatomized the data security sharing and access control mechanism based on blockchain and structured occupational therapy. The detailed chapter arrangement is as follows: Section 2 introduces research methods and data acquisition; Section 3 is survey result analysis; Section 4 is the discussion; Section 5 is the conclusion.

## 2. Research Methods and Case Background

### 2.1. Case Background

In the face of the global epidemic of the COVID-19 virus, the epidemic prevention and control work involves typical public administration and resource allocation; therefore, this paper takes the COVID-19 epidemic prevention and control as an example to carry out public administration based on blockchain-structured occupational therapy on resource allocation methods. Epidemic prevention and control are faced with a new organizational system, new tasks, new environment, and new requirements. Its planning and design, organizational leadership, system construction, business instructions, communication and coordination, material preparation, as well as the collection, identification, and archiving need to start from scratch, and the preliminary work seems rushed and passive. Public administration and resource allocation are coordinated and coordinated by multiple systems, departments, departments and professions, and joint prevention and control, and group prevention and group governance are required. Since the outbreak of the new coronavirus, according to the needs of local epidemic prevention and control work, many leading groups of epidemic prevention and control have been quickly established in various regions to undertake important professional functions of epidemic prevention and control in the region. Its member units include publicity, health, public security, civil affairs, emergency management, big data management, transportation, commerce, economy and letter, market supervision, airports, railways, civil aviation, and customs.

The blockchain can effectively realize the data integration of the whole process and all departments, show the whole picture of the data, and realize the traceability of the whole process. In the process of traditional material access and dispatch, the logistics, warehousing, distribution, and delivery of materials flowing from the distribution end to the end user have not been effectively integrated. Due to the limitations of the development stage, the diversity of needs, and the imperfect information resource governance mechanism, it is difficult to trust each other between departments, the scope of information sharing is not wide, the update of information resources is not timely and inconsistent, and business collaboration is difficult, etc. The problem has been difficult to solve effectively, so it is necessary to find a more reasonable operation mode for the governance of basic information resources of public administration departments. The asymmetric encryption technology in the blockchain can meet the needs of information ownership verification and information security. Its distribution effect can be imagined by combining this fragmented resource allocation process with a public organization [9]. However, the application of blockchain technology can realize the real-time operation of all information of resource allocation on the chain. Not only the logistics information of materials flowing from the distribution terminal to the user can be seen in the whole process but also can be displayed in a panoramic view by means of text, voice, pictures, or videos. Information such as material name, quantity, model, and weight, whether it is the distribution end or the user end, has a predictable distributed ledger that can be consulted.

### 2.2. Data Quality Collaboration Model

With the help of this blockchain technology, the dissemination of various information and events in the process of public administration can cross the middle layers and quickly reach the decision-making layer and the grass-roots level, so that information can be quickly reflected. With the application of blockchain technology, all information on resource allocation will be recorded in the chain, and any changes made by anyone will be directly known to everyone, thus effectively forming a restriction mechanism. In addition, due to the point-to-point transmission, there is no distortion, distortion, change, and other problems in the information transmission process. In a word, blockchain revolutionizes the hierarchical leadership of traditional resource allocation, narrows the distance between superiors and subordinates, spreads information more smoothly, and handles things more efficiently, making the final formation of resource allocation more flat. For the internal relationship of resource allocation, applying the empowerment function of blockchain technology to allocate the corresponding rights to the corresponding stakeholders can significantly reduce the cost of collaboration and management within resource allocation. For example, the system bill of resource allocation can be updated synchronously through blockchain technology, and any changes in the account will be known to stakeholders. This makes the accounts more open and transparent, protects the interests of stakeholders, and reduces the possibility of insiders tampering with the accounts [10].  Figure 1 shows the data quality collaboration model for public administration and resource allocation based on blockchain and structured occupational therapy.

The transformative significance of blockchain technology is that, as a general technology, it must obtain the unanimous consensus of relevant parties before it can be widely used in different fields based on the inapplicability of the governance system. The rise of blockchain has raised new governance requirements and challenges for open and distributed resource allocation, and diversified consensus mechanisms have become new rules and new ways to solve coordination problems. The identity credibility system can authoritatively record and evaluate the credibility of the subjects and their behaviors of data sharing, opening, access, and use. A data sharing and open application achievement supervision platform can build a basic industry transformation situation system driven by data users, data value output, and data value distribution. As a combined innovation of a series of technologies, the release of its value depends more on the specific needs of the application environment, and the related cross-domain collaboration and the degree of digitization of the application environment have become the prerequisites for the realization of change. Furthermore, for organizational change, blockchain still has limitations in reducing transaction costs and improving transaction efficiency under complete contracts. Incomplete contract objectively requires the application of blockchain to sacrifice a certain degree of uncertainty in order to constitute the application premise of complete contracts.

### 2.3. Standard Management Methods for Multiparty Collaboration

Blockchain structured occupational therapy refers to the combination of resource allocation and blockchain, and the use of blockchain technology to solve various specific problems such as incomplete information, soaring transaction costs, and the existence of intermediaries in the development process of resource allocation. The goal of blockchain structured occupational therapy is to upgrade and transform resource allocation, so as to transform resource allocation from low-added value to high-added value, from high energy consumption to low energy consumption, and from extensive to intensive. In the original trust system of resource allocation, state agencies or large enterprises provide mutual trust endorsements, so that the trust system within resource allocation can be maintained, but it is subjective and relatively fragile. As shown in Figure 2, information encryption technology and the use of information traceability technology can achieve the reconstruction of the trust system. In the process of resource allocation development, the refined division of labor also makes the resource allocation chain lengthy. The precise poverty alleviation system established by modern blockchain technology is different, because it has the function of information symmetry in this system. At the same time, this structured occupational therapy also has the characteristics of various innovative application modes of computer technology, including encryption algorithms. The tightness of the resources and the effective allocation of resources are completed, so as to achieve high-quality integration of the resource distribution chain.

Based on blockchain technology, the following changes will occur in the resource allocation process: first, before the start of business, public administration can negotiate various treaties for allocation and sign allocation agreements, agreeing on the type, quality, price, and delivery of allocated resources, methods and dates, offers, insurance, returns, liability for breach of contract, etc. Then, the public administration writes the agreed contract into code, uploads it to the blockchain, and completes the node verification of the entire network. Once the object places an order for a certain resource, the triggering conditions are met, and a series of subsequent outbound, delivery, and financial accounting processes are carried out and can be executed automatically by smart contracts [11]. In this way, the transaction can be completed without the review of the management personnel, the process is greatly simplified, and the payment will be automatically transferred to the public administration account according to the contract, which saves all the links for the recovery of the payment, not only reduces the management cost but also conducive to public administration to do cash budget management. Second, automated and electronic operations reduce the possibility of manual operations and reduce the risk of internal control in public administration. In addition, from the time the object is placed, the public administration can update the distribution data from the database in real time, and all the information from the stock out, delivery, to the object receipt, payment, etc. can be queried and monitored in a timely manner.

## 3. Results and Analysis

### 3.1. Public Administration Mechanism Based on Blockchain and Structured Occupational Therapy

As an embedded programmed contract, a smart contract ensures that both parties can reach a transaction without a centralized organization. As a set of automatically executed code programs, smart contracts can be entered, executed, and ended on the blockchain platform as long as the two parties to the transaction reach a consensus on the program content. This avoids the possibility of disputes arising from the modification of the contract by one of the two parties at the technical level. As long as the electronic contract retained by both parties is processed and then proofread, if it is inconsistent, it proves that the contract has been modified. In the bureaucratic system, higher-level organizations and decision-makers expect their own instruction to be effectively communicated, which includes two meanings: one is the efficiency of instruction transmission. Of course, they expect that grassroots agents can fully implement their own instructions, truly upload and issue them, exert the effect of instructions, and realize policy expectations. However, in the process of uploading and releasing, how to ensure that the will of the upper level is fully understood by the lower-level organization, and the effective implementation and execution are not out of shape, but also to strengthen, and even to prevent the phenomenon of policy idling. In other words, the existing communication system to a large extent only improves the transmission efficiency of information instructions and does not effectively supervise the execution quality of information instructions.

Table 1 shows the blockchain characteristics in the public administration and resource allocation of the prevention and control of COVID-19 epidemic. The peer-to-peer network (P2P) is the underlying network architecture of the entire blockchain, which is a peer-to-peer network architecture that does not have a central server and relies on user group nodes for information exchange. Each node in the network is both a client and a server, and can serve as a server to other node provides services. Each computer node is directly connected, and many nodes together form an end-to-end network. The data cannot be concealed, and at the same time, the cost of postmodification of the data saved by blockchain technology is very high, so that the authenticity of the data can be technically guaranteed. Public character prevails over self-interested motives, and public managers may choose a behavior that focuses on public interests and try to avoid unreasonable distribution of social values in the process of exercising public power. Using the network to build a public administration and resource allocation solves the network bottleneck problem, ensuring that the blockchain is a distributed decentralized system without central equipment, which greatly improves resource utilization. The public key and private key of the asymmetric encryption algorithm are used to identify the owner to disseminate information and realize mutual trust between the transaction parties in the blockchain system [12].

The three main subjects of social resource allocation have their own functions in different social fields, and at the same time, they learn from and penetrate each other. Where the functions of government, market entities, and private entities all play a role to a certain extent at the same time, but the effect of any one entity acting alone is not significant enough, the three entities will be combined according to a certain way of division of labor. Therefore, the government takes financial subsidies, while market entities invest in shares, or social entities provide professional services and charge appropriate fees to form government guidance, supervision, and financial subsidies, which are responsible for managing the three-dimensional cooperation model. Different social resource allocation subjects use different ways in social resource allocation [13]. Market subjects mainly use the law of value and market mechanism, government subjects mainly use legal levers and administrative means, and nongovernmental subjects mainly use customs, customs, morality, and public opinion. Due to the differences in the social foundations, ideological origins, value orientations, and forms of expression of these three types of rules, differences, and conflicts often arise in understanding and application, making social resource allocation structures obstacles and difficulties in mutual cooperation.

### 3.2. Resource Allocation Method Based on Blockchain and Structured Occupational Therapy

The blockchain stores data through a chain block structure with internal timestamps to generate time series for data, and any two blocks are associated with cryptographic methods, which can be traced back to the data information of any block; thus, it has strong traceability and verifiability. Suburbs with vast administrative areas undertake more tasks of infrastructure and public services than central urban areas, such as rail transit, municipal roads, rural roads, bridges, water conservancy facilities, sewage treatment facilities, garbage treatment facilities, large-scale greening, environmental governance, financing, construction and operation management of water supply facilities, power supply facilities, and gas supply facilities [14]. The identity chain is constructed by a system of data integration, confirmation, sharing, and contribution based on individual identity based on the combination of blockchain and big data, forming a business application scenario based on individual identity data. They grasp the most urgent and most in-demand public service problems, rationally allocate government resources, and mobilize social resources to reduce costs and improve allocation efficiency. Suburban financial resources are largely consumed in infrastructure and urban construction projects, and there is a lot of pressure on spending growth in science, education, culture, health, and social livelihood (Figure 3).

Any subject in the system can verify the public ledger, and there is no single subject in the system that can specifically control the public ledger. In contrast to traditional centralized or centralized public decision-making, the public ledger of such management and decision-making activities provided by blockchain technology has distributed data storage and point-to-point transmission and consensus mechanisms in the precise poverty alleviation system. The blockchain-structured occupational therapy uses the point-to-point transmission mode and utilizes the characteristics of decentralization to speed up the turnover of funds and commodities and strengthen the resource allocation chain. The mechanism of this information symmetry lies in the fact that scientists use mathematical principles to establish machine credit in the system, which fundamentally subverts the information asymmetry drawbacks of the traditional centralized and centralized management model [15]. This information asymmetry of any other subject other than the transaction subject is the source of various irregular transactions. Any economic behavior of traditional centralized management is asymmetric information, resulting in difficult to judge government costs.

In the blockchain technology environment, the parties to the transaction automatically input data through the Internet of Things, mobile terminals, or artificial intelligence devices, etc. and record and save the data with the cryptographic technology of the blockchain. If party A generates a pair of keys and discloses one of them to other parties as a public key; party B who obtains the public key uses the key to encrypt the confidential information and then sends it to party A; the encrypted information is decrypted by another private key. Different from the usual client-server network architecture, in the network environment, thousands of computers connected to each other are in a peer-to-peer position. In the field of public administration, since public power assumes the function of authoritatively distributing the value of the whole society, if the public manager in charge of public power lacks the restraint of public spirit and external institutions, it may use various public resources to form own vested interests. Facing the temptation of interests, the public character and self-interest motives of public managers are always in a state of intense competition. The public managers whose self-interest motives prevail, the driving force of their actions is the maximization of personal interests. This is the most fundamental reason for the formation of vested interests of public managers, and it is also the most difficult motivation for public managers to overcome and prevent.

## 4. Discussions

### 4.1. Role of Distributed Ledger to Increase the Information Symmetry of Public Administration Activities

Based on a distributed peer-to-peer network, blockchain allows participants to join freely or authorized, thereby establishing a social governance system of collective participation and collective maintenance. Through the consensus mechanism, all participating nodes on the blockchain can reach a consensus on transactions or behaviors, thereby establishing a new order in the digital society. As shown in Table 2, the blockchain records the data of the whole network, the whole process, and the whole transaction, and all the data is jointly owned by all the nodes of the whole network, the government affairs information is more transparent, and the data writing behavior is more traceable, so as to realize the participation of all members in social governance, and the full participation of all members in a new mechanism for consensus and full supervision [16]. Blockchain technology solves the technical obstacles of previous smart contract implementation and has the advantages of decentralization, nontampering, process transparency, traceability, etc., so that the decentralized ledger function of blockchain can be used to create, confirm, and transfer various types of assets and contracts. The centralized ledger model, which becomes the center to maintain and manage the ledger, becomes the key to management. Blockchain technology can allow data to be shared in a new type of information trading market and even the utility of sharing data. Blockchain provides a new idea and method for coordinating these services and is a true digital technology-driven approach to realizing a credit society.

Integrity supervision of public administration is not only an institutional project but also a technical practice. The technical characteristics of blockchain, such as decentralization, data transparency, security and reliability, privacy protection, nontampering, traceability, and detrust, are very important to the improvement of the system and mechanism of promoting clean government supervision and the improvement of technical governance efficiency provide important support, and the two are closely related in internal logic. The blockchain can incorporate the supervision power of citizens and society into the integrity supervision system, so that the supervision of power can evolve from single-center supervision to multicenter supervision, and all public powers can be supervised. Second, the essence of blockchain is a distributed ledger, which ensures the sharing and disclosure of information and data. Third, the public key of the blockchain plays the function of information disclosure in the determination, display, control, and regulation of power, which helps to open the black box of major public affairs and major project decision-making. Therefore, blockchain technology is logically related to the democratization of clean government supervision. The blockchain data layer and network layer technology jointly ensure that the transactions cannot be tampered with. Once the information is tampered, it will broadcast and notify all participants and will lead to the failure of information tampering.

An important application of the antitampering feature of blockchain in the social governance of data is to ensure the security and reliability of historical data. The traditional center-periphery structure, the center enjoys the convenience of observing the entire structure due to its central position, and this convenience also provides the center with a unique global perspective. The center of the structure can see all the transactions in the structure and then master the complete ledger, which is generally believed that one of the advantages of this model is that it is convenient to provide sufficient evidence for dispute arbitration. However, the advantages are also disadvantages. Since the center enjoys the absolute right to process data, this right will be changed due to the opaqueness of the central organization and its data processing process [17]. It is more powerful, which makes the ledger information possible to be tampered with by the center in the direction of its own benefit. Even if the center data is indeed damaged due to objective reasons, the public is more inclined to the cause of human sabotage. In this sense, some specific information randomly generated in blockchain applications is indeed more helpful to protect the privacy of users. However, more importantly, the central agency prefers that similar identifications be unique or as few as possible, and a person's identity card and number must be unique.

### 4.2. Blockchain-Established Special Machine Trust for Resource Allocation

Public administration big data governance has always been the main content of public administration construction. Its purpose requires the management of big data to be centered on the service object and to achieve complete and timely information flow and cross-platform cross-department, cross-field, and cross-platform public administration at all levels and types. Public administration big data is an important part of public administration big data governance, the core content of data governance, and plays an important role in cross-departmental collaboration. Blockchain-established special machine trust for resource allocation based on blockchain and structured occupational therapy is shown in Figure 4. Public administration big data can be divided into two categories: basic information and extended information, that is, the description information of the basic situation of objects required by all public administration departments and the business-specific information corresponding to the interaction activities of citizens, enterprises, and government departments. Although the logistics information of resource allocation can be updated in real time, it is only visible to the sender or recipient, especially resource allocation generally requires a distribution center or a command center to match supply and demand. Therefore, the circulation of information and value in the national governance system is limited by the authority and power of the government, which is unable to achieve direct interoperability. The cryptography principle of blockchain ensures the integrity, consistency, and continuity of data through a consensus mechanism, forming a standard database that is difficult to tamper with.

The blockchain-based open network model for government data sharing can build a consortium chain of government functional departments, a government-oriented public chain for the public, and a public security system based on the sensitivity of the data carrier. It can form a blockchain rope network structure for government data sharing and openness, create a credible government data sharing and open platform, ensure the openness and security of data sharing among various functional departments of the government, and solve the risks associated with big data [18]. It should be pointed out that although the consensus mechanism seems to be an innovation at the technical level, when it jumps out of the limitation of the technical perspective and starts from the perspective of the evolution of resource allocation rules, the blockchain also brings transformative significance at the institutional level. As the population of the central urban area is exported, its management, security, and services are also exported to the suburbs, and most of them are nondividend people who are difficult to find employment. The identity chain project is based on the data related to individual identity to form a system mechanism for the application management, which integrates the security integration, standardized application, effective confirmation, and sharing incentives of individual identity data and business processes.

The core feature of the blockchain formed based on the above mechanism is that all transaction information is stored on the chain. It is theoretically impossible to achieve; at the same time, any participant in the network can store the entire blockchain, thus forming a distributed storage, and the collapse of any node will not affect the normal operation of the entire network. With the help of the decentralization and nontampering characteristics of blockchain technology, which is easy to trace back, a public decision-making responsibility mechanism for the self-organized operation of the government service platform under the assistance of the government is constructed [19]. This requires changing the practice of mandating the openness of data and information, and instead building a data platform, supervising the operation, and handling disputes. For example, each subject is required to perform operations on the mastered data and record it in the blockchain. Public agencies are only responsible for building, maintaining, and supervising the operation of blockchain platforms. Through blockchain technology, the access information and utilization information of each data set will be recorded and sealed, thus ensuring the security of data information and protecting privacy, and thus providing various subjects with tracking and accountability for other people who use the data.

### 4.3. Data Security Sharing and Access Control Mechanism in Public Administration and Resource Allocation

Credit-based resource allocation mostly requires credit endorsement from third-party institutions. In the traditional state governance system centered on the government, bilateral or multilateral interactions rely on government departments as trusted intermediary organizations for coordination and are constrained by this administrative system [20]. As a highly centralized system, government departments hold a large amount of high-density and high-value information, and only a small amount of information is scattered in the hands of other stakeholders. Therefore, all information is gathered in the distribution center, and the information between the material issuer and the end user at the distribution end is extremely asymmetric, which easily induces the intermediate link to exercise discretion and adapt to the distribution object, distribution method, and distribution time of the material. Instead, blockchain builds a peer-to-peer distributed peer-to-peer network among different stakeholders through structured occupational therapy, and updates of information will be reflected and confirmed in each database in a timely manner (Figure 5). The consensus mechanism urges each governance body to abide by a unified agreement and without a strong third-party organization to coordinate, supervise, and highly decentralized decision-making powers, reach agreement or consensus on the validity of data, and perform their own responsibilities and spontaneously coordinate. Form an ordered self-organizing network.

The decentralization of the blockchain is conducive to building an open, transparent, green, fair, and efficient cross-departmental and cross-level emergency management collaboration platform. Any relevant government department can rely on the platform to obtain high-credibility data in real time, and synchronously record, upload, and store work information on the platform, providing an information foundation for collaboration and cooperation between government departments. The decentralized management collaboration platform can realize cross-departmental and cross-regional maintenance and utilization of government data, promote business collaboration, achieve clear instructions, orderly systems, smooth and efficient execution, and improve the integration efficiency of internal government resources. The responsibilities of each department are managed through relevant electronic programs. The algorithm code of the program contains conditions that will trigger the automatic execution of the contract. When the smart contract is uploaded to the blockchain platform, the program will automatically check the relevant events and trigger conditions and meet the conditions. The work will be directly assigned to the relevant departments, and the progress of the work will be monitored in real time. Smart contracts use algorithm code as the standard for responsibility delimitation, which can effectively prevent buck-passing and overcome laziness. At the same time, the automatic triggering and execution of algorithms can reduce manual approval and can also improve the degree of automation of government work and the quality of public services [21].

The essence of social governance is the government's service and management of the society. The government improves and protects people's livelihood through social governance, achieves a trust relationship between the government and society, and forms a social consensus, thereby promoting social development. Therefore, social public trust is a major issue in social governance. Blockchain can use its advantages of information sharing, data traceability, authenticity and reliability of data, and immutability to improve the transparency of public information to the public, so that the public sector can get rid of the crisis of public trust [22]. Structured occupational therapy can build a blockchain-based government trust model, build a reliable environment and mass base for government trust, and use blockchain tools to rationally decentralize and detrust, so as to fundamentally get rid of the public trust crisis. Based on the consensus mechanism of the distributed structure, the blockchain will replace the traditional trust structure endorsed by third-party credit institutions with decentralized system trust, and establish a transparency, immutability, traceability, and distributed storage based on the data itself. The new credit reporting system enhances peer-to-peer trust by reducing information asymmetry. The distributed ledger built by blockchain based on cryptography improves the security and effectiveness of data transmission, thereby solving information security and trust issues in volunteer service.

## 5. Conclusions

In order to explore the public administration and resource allocation based on blockchain and structured occupational therapy, this paper takes the public affairs in the prevention and control of the COVID-19 epidemic as an example to conduct research. This study discussed the public administration mechanism based on blockchain and structured occupational therapy, established a resource allocation method based on blockchain and structured occupational therapy, fathomed the role of the distributed ledger established by blockchain to increase the information symmetry of public administration activities, proposed a blockchain-established special machine trust for resource allocation, and finally, anatomized the data security sharing and access control mechanism based on blockchain and structured occupational therapy. Blockchain can use its advantages of information sharing, data traceability, authenticity and reliability of data, and immutability to improve the transparency of public information to the public, so that the public sector can get rid of the crisis of public trust. The asymmetric encryption technology in the blockchain can meet the needs of information ownership verification and information security. The consensus mechanism urges each governance body to abide by a unified agreement and without a strong third-party organization to coordinate, supervise, and highly decentralized decision-making powers, reach agreement or consensus on the validity of data, and perform their own responsibilities and spontaneously coordinate. The blockchain revolutionizes the hierarchical leadership method of traditional resource allocation, shortens the distance between superiors and subordinates, makes information dissemination more fluent, and handles things more efficiently, making resource allocation ultimately form a flatter organization structure. In the original trust system of resource allocation, the blockchain and structured occupational therapy realizes the reconstruction of the trust system by preventing information tampering, using information encryption technology, and using information traceability technology. The results of this paper provide a reference for further research on the public administration and resource allocation based on blockchain and structured occupational therapy.

## Figures and Tables

**Figure 1:** Data quality collaboration model for public administration and resource allocation based on blockchain and structured occupational therapy.

**Figure 2:** Standard management methods for multiparty collaborations in public administration and resource allocation based on blockchain and structured occupational therapy.

**Figure 3:** Resource allocation method in public administration and resource allocation based on blockchain and structured occupational therapy.

**Figure 4:** Blockchain-established special machine trust for resource allocation based on blockchain and structured occupational therapy.

**Figure 5:** Data security sharing and access control mechanism in public administration (a) and resource allocation (b) based on blockchain and structured occupational therapy.

**Table 1:** Blockchain characteristics in the public administration and resource allocation of the prevention and control of COVID-19 epidemic (note: +: have; -: does not have).

Item	Distributed ledger	Asymmetric encryption	P2P transmission	Smart contract	Consensus mechanism
Publicity	+	-	-	-	-
Hygiene and health	+	+	-	+	-
Public security	+	+	-	+	+
Civil affairs	-	+	+	-	+
Emergency management	-	+	+	+	+
Big data management	+	-	+	-	-
Transportation	+	-	+	+	-
Commerce and economy	-	-	+	-	-
Market supervision	-	-	+	+	+
Customs	-	-	+	+	+
Planning and design	-	+	-	+	-
Organizational leadership	-	+	+	-	-
System construction	+	-	-	-	+
Material preparation	+	+	-	+	-
Airports	+	-	-	+	+
Railways	-	+	+	+	-
Civil aviation	+	-	+	+	+
Communication	-	-	-	-	-
Environmental governance	+	-	+	-	+
Business instructions	-	+	-	-	+
Logistics and delivery	-	+	+	-	+

**Table 2:** Role of distributed ledger to increase the information symmetry of public administration activities.

Item	Network	Process	Method	Model
Publicity	[1]	A	(3)	*d*
Hygiene and health	[3]	B	(5)	*d*
Public security	[5]	D	(4)	*a*
Civil affairs	[3]	A	(1)	*c*
Emergency management	[4]	B	(2)	*a*
Big data management	[5]	B	(3)	*c*
Transportation	[2]	A	(2)	*d*
Commerce and economy	[2]	A	(5)	*a*
Market supervision	[3]	C	(3)	*a*
Customs	[1]	A	(1)	*d*
Planning and design	[1]	D	(1)	*b*
Organizational leadership	[4]	C	(5)	*a*
System construction	[3]	B	(4)	*b*
Material preparation	[5]	C	(4)	*c*
Airports	[2]	D	(2)	*b*
Railways	[2]	A	(2)	*a*
Civil aviation	[4]	A	(3)	*d*
Communication	[5]	B	(1)	*b*
Environmental governance	[3]	D	(1)	*a*
Business instructions	[2]	C	(4)	*b*
Logistics and delivery	[1]	A	(5)	*d*

Note: [1]: central server; [2]: user group node; [3]: client server; [4]: regulatory platform; [5]: control group node; A: security integration; B: standard application; C: effectiveness confirmation; D: sharing incentives; (1): distributed ledger technology; (2): asymmetric encryption algorithm; (3): peer-to-peer transmission; (4): smart contract; (5): consensus mechanism; *a*: traceable time in chronological order; *b*: distributed decentralized structure; *c*: coordination intelligence for information security; *d*: data authenticity and reliability.

## Data Availability

The data used to support the findings of this study are available from the corresponding author upon request.
